The article "The Application of Virtual Reality Technology in Sports Psychology: Theory, Practice, and Prospect" was published in 2022. Journal: Comput Intell Neurosci.

# The Application of Virtual Reality Technology in Sports Psychology: Theory, Practice, and Prospect

**DOI:** 10.1155/2022/5941395

**Published:** 2022-08-11

**Authors:** Yu Liu, Shuang Li, JunRu Guo, GuoLiang Chai, ChunMei Cao

**Affiliations:** ^1^Department of Psychology, Guizhou Minzu University, Guiyang 550025, Guizhou, China; ^2^College of Physical Education, Guizhou University, Guiyang 550025, Guizhou, China; ^3^Division of Sports Science and Physical Education, Tsinghua University, Beijing 100084, Beijing, China

## Abstract

Once virtual reality technology (Virtual Reality, VR) came out, it has received a lot of attention; in recent years, it has been widely used in the study of psychology. Because it can improve the ecological validity of experimental research, the level of conditional control, reproducibility, and avoid the dangers of field operations, it has been introduced into the field of psychology by many researchers. Compared with traditional sports psychology research methods, virtual reality technology has the characteristics of multiperception, immersion, interaction, and imagination to get a better, more realistic feel and increase people's interest in sports. Taking the application of virtual reality technology in table tennis teaching in colleges and universities as an example, this study aims to review the application of virtual reality technology in sports psychology; summarize the theory, practice, and prospect of the application of virtual reality technology in sports psychology; and add new content to the research of sports psychology. It aims to review the principles, characteristics, and application of virtual reality technology in sports psychology; summarize the advantages and disadvantages of the application of virtual reality technology in sports and point out the problems that need to be paid attention to when using this method; explore the application of virtual reality technology in sports psychology; and add new content to the research of sports psychology.

## 1. Introduction

Virtual reality (VR) is a representative of high-tech products in the Internet era. The computer system simulates the human feeling through programming, and the virtual world that presents it in real time is the virtual environment [1]. With the continuous development of computer hardware and the continuous development of software programming technology, virtual reality technology has gradually been applied to medical treatment, sports, education, teaching, psychotherapy, etc. These features of virtual reality can provide students with an interesting teaching environment, provide patients with a variety of treatment methods, and provide new sports methods for physical exercise, which has penetrated people's daily lives in many ways. Based on virtual reality technology, this article studies the development of competitive sports simulation applications [2].

The article "The Application of Virtual Reality Technology in Sports Psychology: Theory, Practice, and Prospect" was published in 2022. Journal: Comput Intell Neurosci.

At present, various new technologies and methods have been widely adopted in the field of psychology for research, such as event-related potential (ERP) and functional magnetic resonance imaging (fMRI). In recent years, foreign researchers have used virtual reality technology to study psychology and achieved fruitful results. In psychological research, the virtual environment created by virtual reality technology is not only a revolutionary change in the replication, simulation, and representation of the external world in the real world, but also a new research tool and research paradigm.

VR technology has received great attention from various fields at the beginning, but due to its expensive development cost, it is generally only developed for special purposes. With the rapid development of computer science and artificial intelligence technology [3], VR technology can be said to be changing with each passing day, not only the great improvement in “3I” characteristics, but also the accompanying introduction of personal consumer VR products [4], which makes the popularization and application of VR technology possible [5]. At present, VR technology is being widely used in public safety, industrial design, medicine, planning, transportation, culture and education, and other industries and departments [6]. At the same time, in the field of psychology, more and more researchers try to apply VR technology to experimental research, psychological assessment, and clinical psychotherapy [7]. Generally speaking, according to the different presentation methods, VR is divided into nonimmersive (mainly presented directly on a computer screen) and immersive (such as helmet-based and cave-based) VR systems. Nonimmersive VR systems are less expensive, but their nonimmersive nature makes them more suitable for experiments that require simple reactions [8]. On the contrary, the immersive VR system can bring a more realistic and complex physiological and psychological experience to the individual, which is the mainstream of VR research and application in recent years [9]. This article aims to review the principles, characteristics, and application of virtual reality technology in sports psychology; summarize the advantages and disadvantages of the application of virtual reality technology in sports and point out the problems that need to be paid attention to when using this method; discuss the application of virtual reality technology in sports psychology; and add new content to the research of sports psychology.

The article "The Application of Virtual Reality Technology in Sports Psychology: Theory, Practice, and Prospect" was published in 2022. Journal: Comput Intell Neurosci.

## 2. Virtual Reality Technology and Related Research Progress

### 2.1. Virtual Reality Technology

Virtual reality (VR) is a new type of technology that integrates simulation technology, multimedia technology, sensing technology, network, and other technologies. Using computer graphics, simulation technology, multimedia technology, artificial intelligence, network technology, parallel processing, and multiparameter environment perception to simulate human vision, hearing, touch, and other sensory organs, people are immersed in the virtual world. In addition to instant interaction through language and gestures, it creates a multidimensional data space for people with broad application prospects. The actual policy of simulated VR is to process sensor data with the help of a series of sensor-integrated equipment, build a VR virtual environment based on fusion information, and finally realize the mutual interaction between the real world and the virtual space and exert its maximum value.  Figure 1 shows the multisensing VR interaction model [10].

The virtual environment generator, the input system, and the output system are the three structures that constitute the VR sports simulation system. The specific contents are shown in Figure 2 [11]. Among them, the user system, high-performance computer, simulation manager, and 3D model database together constitute a virtual environment generator; effect generator and signal converter together constitute an output system; converter, glove input conversion, position and direction tracker, data glove, etc [12]. Together, they form an input system. With this as the background, the user's feeling of the environment is more realistic, and the natural interaction process between their own feelings and the virtual environment is realized, and there is an immersive feeling. Therefore, there is a wide range of applications for applying virtual reality technology to sports psychology.

### 2.2. Research on Virtual Reality Technology at Home and Abroad

The development law of virtual reality technology is closely related to the growth law of research literature, and the change in the number of studies in virtual reality technology research directly reflects the change in research development. Therefore, the number of research studies on virtual reality technology at home and abroad is one of the important yardsticks to measure its technical application and development. From 1995 to 2019, scholars from 72 countries have published research literature on virtual reality, of which the United States is the highest producing country (1041), followed by the United Kingdom (310), and China ranks third (285), followed by Germany (259), Spain (232), Canada (215), South Korea (215), Italy (206), etc [13] (Table 1). It can be seen that European and American countries are still in a leading position in the field of virtual reality research. My country's virtual reality technology started in the early 1990s. With the rapid development of digital technology and computer systems engineering, virtual reality technology has received great attention. Since 2016, virtual reality has been listed as an emerging frontier industry, which has greatly promoted the research and development enthusiasm of scientific researchers and made the virtual reality market in China more prosperous [14]. We have ushered in a new era, but in terms of the number of national publications, there is still a big gap with European and American countries, which is mainly limited by differences in economic conditions, cultural background, and scientific research capabilities. In general, every year, new countries join the research of virtual reality technology, which can be divided into the following three stages [15]. Development period: since 2012, emerging countries such as Iran, Saudi Arabia, Lithuania, Pakistan, and Jordan have also begun to work on virtual reality research [16].

The article "The Application of Virtual Reality Technology in Sports Psychology: Theory, Practice, and Prospect" was published in 2022. Journal: Comput Intell Neurosci.

The competitive sports simulation system designed this time can simulate the scene in the competitive sports competition, and record the competitive sports actions and data involved in it, so as to judge whether the sports players' actions are standard and target their defects which need improvement [17]. Therefore, the integration of the competitive sports simulation system and VR technology needs to meet the data output and input functions, and it is necessary to ensure that the sports athletes' competitive sports actions are simulated as much as possible on the basis of VR technology, so as to experience the most real and best sports at any time. A reliable competitive sports simulation environment can be created in this way. The system function interaction structure is shown in Figure 3.

## 3. Research Objects and Methods

### 3.1. Research Objects

This research takes the impact of virtual reality technology applied to table tennis teaching in colleges and universities as the research object (Table 2) and selects 97 college students in three parallel classes of the 2018 non-sports major table tennis elective course in a college as the survey object, in order to explore the integration. The application value of virtual reality technology teaching mode in college table tennis teaching is very high.

### 3.2. Research Methods

Literature data method: In order to deeply understand the application of virtual reality technology in table tennis teaching, according to the purpose and content of this research, searches on the Chinese databases: University Library, CNKI database, Wanfang academic database, and English databases: Web of Science and Science Direct, were organized and relevant data were summarized, and scientific literature visualization analysis software was used to conduct in-depth excavation of the included literature [18].

The article "The Application of Virtual Reality Technology in Sports Psychology: Theory, Practice, and Prospect" was published in 2022. Journal: Comput Intell Neurosci.

Questionnaire survey method: In this study, 97 college students from three parallel classes of table tennis elective courses in a university were selected as the subjects of the questionnaire to investigate their interest in sports situations and the autonomous learning of college students' sports [19].

The main experimental steps in this article are as follows:

1. The 97 college students selected in this article are divided into three groups according to the three types of traditional courses, virtual reality teaching courses, and video teaching courses according to different departments, and the number of the three groups is 34, 32, and 31, respectively. The three groups of faculties are social development and public administration, the School of Arts and the College of Education, with the traditional course group and video course group as the control group of this article, and the virtual reality course group as the experimental group of this article.
2. After a one-semester table tennis class, a questionnaire survey is conducted on the passage of three groups of experiments by developing a corresponding questionnaire.
3. Using mathematical statistics software, the results of the questionnaire are first tested for reliability and validity, so as to verify the scientific nature of the questionnaire and show that the experimental results can be used for research.
4. The students' independent learning ability in the questionnaire results, the consistency of students' interest in sports situations, and the learning effect of virtual reality teaching classes are analyzed, so as to explore students' interest in virtual reality teaching and prove the application value of the integrated virtual reality technology teaching mode in the teaching of table tennis in colleges and universities.

### 3.3. Description of Survey Tools

#### 3.3.1. FK Algorithm

The movement is divided into forward movement and reverse movement. FK is the abbreviation of forward kinematics, that is, forward dynamics; IK is the abbreviation of inverse kinematics, that is, inverse dynamics. The skeleton of the human body is composed of many link chains that are grouped in a hierarchical manner, including hierarchical structure joints or chains, motion constraints, and effectors, which drive all parts to move simultaneously [20].

The article "The Application of Virtual Reality Technology in Sports Psychology: Theory, Practice, and Prospect" was published in 2022. Journal: Comput Intell Neurosci.

Forward dynamics considers that child joints will follow the motion of parent joints, and child joints can move independently without affecting the state of parent joints. Human motion is taken as an example, as shown in Figure 4.

The advantage of forward dynamics is that the calculation is simple and the calculation speed is fast, since it involves naturally coordinated movements. When applied to the VR motion capture industry, users need to wear motion capture devices in each skeleton branch, which is inconvenient to use.

#### 3.3.2. IK Algorithm

Take the action of hitting the ball as an example: if we know the starting position, final position, and path of the ball, then the rotation of the bowler's arm, etc. can be calculated automatically according to inverse kinematics [21]. The inverse kinematics method relieves the tedious work of the forward kinematics method to a certain extent and is one of the best ways to generate realistic joint motions [22].

Since inverse dynamics can solve the positioning problem, the IK algorithm can be applied to VR motion capture technology and gesture recognition technology [23]. Motion capture technology is taken as an example to illustrate the specific implementation process in Figure 5:

Motion capture technology uses specialized sensors called trackers to record the movement of an athlete. Then, we can use the recorded data to generate animation motion [24].

#### 3.3.3. PNP

PNP is precisely a problem; the PNP problem was proposed by Fisher and Bolles in 1981 [25]. PnP translates as plug and play. The specific expression of the PNP problem is as follows: the distance between any two feature points in a given *n* feature points and the angle formed between the two feature points and the optical center are known to solve the distance between each feature point and the optical center. There are many ways to solve the PNP problem, which can be roughly divided into two categories, noniterative algorithms and iterative algorithms:

When the iterative algorithm is applied to solve the PNP problem, it is derived based on the assumption that there is no image noise. In order to overcome the influence of noise and improve the accuracy of pose calculation, the PNP iterative algorithm is often used to solve the pose information [26]. The main idea is to further express the PNP problem as a constrained nonlinear optimization problem. A numerical solution can measure the relative pose of the target. The optimization variable space of this processing method is the *N* + 6 dimension (*N* is the number of point features), the amount of iterative calculation is large, and it is affected by the accuracy of the initial value solution, so the algorithm usually converges to the local minimum or converges to the wrong solution, rather than the global minimum [27]. P3P is taken as an example and illustrated in Figure 6.

The article "The Application of Virtual Reality Technology in Sports Psychology: Theory, Practice, and Prospect" was published in 2022. Journal: Comput Intell Neurosci.

As shown, *O* is the optical center of the camera; the lengths between the three feature points *A*, *B*, and *C* of the target and the optical center *O* are *x*, *y*, and *z*, respectively; and the angles between the three known lines are *α*, *β*, *γ*, |*AB*| = *c*, |*AC*| = *b* |*BC*| = *a*. *α*, *β*, *γ* and *a*, *b*, *c* can be used to solve *x*, *y*, and *z*: this is the P3P problem.

The number of feature points in the P3P problem is only 3, and the non-iterative algorithm can be used directly. The equation is described as follows:

(1) $$\begin{array}{c} x^{2}+y^{2}=2xy\;\cos\;\alpha =c^{2},\\ x^{2}+z^{2}=2xy\;\cos\;\beta =b^{2},\\ x^{2}+z^{2}=2xy\;\cos\;\beta =b^{2}. \end{array}$$

Suppose *A*′, *B*′, and *C*′ are the points of *A*, *B*, and *C* on the imaging plane of the camera, respectively; then, after obtaining *x*, *y*, and *z*, using the coordinates of *A*′, *B*′, *C*′, according to the camera's imaging relationship, the coordinates of the feature points can be solved in the camera coordinate system. The PNP algorithm can be applied to VR positioning technology, such as infrared optical positioning technology, to obtain pose information [28]. The specific implementation process is that the camera obtains the image of the target object, and then extracts the feature points in the image; then, the PNP algorithm is used to obtain the coordinates of the feature points in the camera coordinate system; and finally, the information of the feature points in the world coordinate system is obtained as shown in Figure 7.

#### 3.3.4. POSIT Algorithm

In fact, the POSIT algorithm is one of the iterative algorithms for the PNP problem mentioned above [29]. First, the initial value of the pose parameters of the three-dimensional object (POS, Pose from Orthography and Scaling algorithm) is obtained through the relationship between orthogonal projection and size transformation [30]. With the new pose measurement parameters, the POS algorithm is re-run, after repeated iterations, until the required accuracy is met in an algorithm flow.

Suppose the attitude to be sought, including the rotation matrix *R* and the translation vector *T*, are

(2) $$\begin{array}{c} R=\left[\begin{array}{ccc} R_{11} & R_{12} & R_{13}\\ R_{21} & R_{22} & R_{23}\\ R_{31} & R_{32} & R_{33} \end{array}\right]\\ =\left[\begin{array}{c} R_{1}^{T}\\ R_{2}^{T}\\ R_{3}^{T} \end{array}\right],\\ T=\left[\begin{array}{c} T_{x}\\ T_{y}\\ T_{z} \end{array}\right]. \end{array}$$

The perspective projection transformation is

(3) $$\begin{array}{c} x=\frac{f}{Z_{c}}X_{c},\\ y=\frac{f}{Z_{c}}Y_{c}. \end{array}$$

(*x*_*c*_, *y*_*c*_) are the coordinates of the image coordinate system in millimeters.

The article "The Application of Virtual Reality Technology in Sports Psychology: Theory, Practice, and Prospect" was published in 2022. Journal: Comput Intell Neurosci.

(*X*_*c*_, *Y*_*c*_, *Z*_*c*_) are the coordinates of the camera coordinate system in millimeters.

The *f* in the above formula is the focal length of the camera, and its specific value is not important. What is important is the ratio between *f* and *x* and *y*. This ratio can be obtained according to the *f*_*x*_ and *f*_*y*_ of the parameter matrix in the camera. In the actual operation, *f* = 1 can be directly set, but the corresponding *x* and *y* should also be set proportionally. For example, for a camera with internal parameters [*f*_*x*_, *f*_*y*_, *u*_0_, *v*_0_], if the position of a pixel is (*u*, *v*), the corresponding *x* and *y* should be

(4) $$\begin{array}{c} x=\left(u-u_{0}\right)\frac{f}{f_{x}},\\ y=\left(v-v_{0}\right)\frac{f}{f_{y}}. \end{array}$$

Suppose a point in the world coordinate system is (*X*_*w*_, *Y*_*w*_, *Z*_*w*_), then

(5) $$\begin{array}{c} \left[\begin{array}{c} Z_{c}x\\ Z_{c}y\\ Z_{c} \end{array}\right]=\left[\begin{array}{c} fX_{c}\\ fY_{c}\\ Z_{c} \end{array}\right]\\ =\left[\begin{array}{c} fR_{1}^{T}\\ fR_{2}^{T}\\ R_{3}^{T} \end{array}\begin{array}{c} fT_{x}\\ fT_{y}\\ T_{z} \end{array}\right]\left[\begin{array}{c} X_{w}\\ Y_{w}\\ \begin{array}{c} Z_{w}\\ 1 \end{array} \end{array}\right]. \end{array}$$

Dividing both sides by TZ gives

(6) $$\begin{array}{c} \left[\begin{array}{c} wx\\ wy\\ w \end{array}\right]=\left[\begin{array}{c} sR_{1}^{T}\\ sR_{2}^{T}\\ R_{3}^{T}/T_{z} \end{array}\begin{array}{c} sT_{x}\\ sT_{y}\\ 1 \end{array}\right]\left[\begin{array}{c} X_{w}\\ Y_{w}\\ \begin{array}{c} Z_{w}\\ 1 \end{array} \end{array}\right], \end{array}$$

in

(7) $$\begin{array}{c} w=\frac{Z_{c}}{T_{z}},\\ W={\left[\begin{array}{ccc} X_{w} & Y_{w} & Z_{w} \end{array}\right]}^{T}.\\ s=\frac{f}{T_{z}}. \end{array}$$

The *i*-th row of *R* represents the coordinates of the unit vector of the *i*-th coordinate axis direction in the camera coordinate system in the world coordinate system; the *i*-th column of *R* represents the coordinates of the unit vector in the direction of the *i*-th coordinate axis in the world coordinate system in the camera coordinate system; *T* is exactly the coordinates of the origin of the world coordinate system in the camera coordinate system. In particular, *T*_*z*_ represents the world. The origin of the coordinate system is the “depth” in the camera coordinate system.

The article "The Application of Virtual Reality Technology in Sports Psychology: Theory, Practice, and Prospect" was published in 2022. Journal: Comput Intell Neurosci.

According to the previous assumption, the “thickness” of the object in the *Z*-axis direction, that is, the *Z*-coordinate variation range of each point on the surface of the object in the camera coordinate system is much smaller than the average depth of the object in the *Z*-axis direction. It is important to note that both “thickness” and “depth” are relative to the *Z* axis of the camera coordinate system. When the origin of the world coordinate system is near the center of the object, it can be considered that the average depth is the *T*_*z*_ component in the translation vector *T*, that is, the average value of *Z*_*c*_ of each point is *T*_*z*_, and the variation range of *Z*_*c*_ is small relative to *T*_*z*_, so it can be believed that *Z*_*c*_ is always near *T*_*z*_, and *Z*_*c*_ ≈ *T*_*z*_.

According to this approximate relationship, we can get

(8) $$\begin{array}{c} w=\frac{Z_{c}}{T_{z}}\approx 1. \end{array}$$

This is our initial iteration value. In this initial state, we assume that all points of the object are at the same depth, and the perspective transformation at this time degenerates into a proportional orthographic projection POS. That is, our iteration starts with a scaled orthographic projection, which is where the POSIT algorithm gets its name.

### 3.4. Issuance and Recovery of Questionnaires

A total of 194 questionnaires were distributed in this experiment, of which 97 were distributed before the experiment and 97 after the experiment. The distribution and recycling of the questionnaires shall be in the form of on-site distribution and on-site recycling. In the process of filling in, if you have any questions about a certain question, you should ask the responsible person in time to ensure the authenticity of the questionnaire. Distribution and recovery: A total of 97 questionnaires were distributed before the experiment, 97 questionnaires were recovered, and the recovery rate was 100%, of which 97 were valid questionnaires, and the effective rate was 100%. After the experiment, a total of 97 questionnaires were distributed, 97 questionnaires were recovered, and the recovery rate was 100%, of which 97 were valid questionnaires, and the effective rate was 100%.

### 3.5. Reliability and Validity Test of the Questionnaire

Reliability test: In order to test whether the test scale is reliable and stable so that the results can reflect the expected goals, in this study, Cronbach's alpha coefficient was used to test the consistency of the questionnaire structure. It is generally believed that the larger the *α* coefficient, the higher the reliability of the questionnaire. When Cronbach's *α* coefficient does not exceed 0.6, the internal consistency reliability is considered unacceptable. When the Cronbach's alpha coefficient is between 0.7 and 0.8, it means that it has a certain degree of reliability. When Cronbach's alpha coefficient is between 0.8 and 0.9, the reliability of the test scale is considered to be very good. In this study, Cronbach's *α* coefficient of 0.7-0.8 was selected as the measurement standard for testing, as shown in Table 3.

The article "The Application of Virtual Reality Technology in Sports Psychology: Theory, Practice, and Prospect" was published in 2022. Journal: Comput Intell Neurosci.

From the reliability test results of the above table, it can be seen that Cronbach's *α* coefficients of each dimension variable of “College Students' Self-directed Learning Scale” and “Sports Situational Interest Scale” are all greater than 0.7, which is consistent with the consistency of the questionnaire structure, indicating that the amount of the scale has good reliability.

Validity test: The validity test is a powerful tool used to measure the content and structure of the scale, as shown in Table 4. In this study, the factor analysis method will be used to test the validity of “College Students' Self-directed Learning Scale” and “Sports Situational Interest Scale.” First, the KMO sample measure and Bartlett's sphere test were applied to see whether the data can be subjected to factor analysis. When the KMO is above 0.90, it means that the validity of the scale is very good; if the KMO is between 0.7-0.9, it means that the validity is acceptable; if the KMO is between 0.5 and -0.7, it means that the validity is average; if the KMO is below 0.5, it means that the validity is acceptable. Validity is not acceptable. At the same time, the significance of the sphere test must be less than 0.05, and the factor analysis is carried out on this basis.

## 4. Research Results and Analysis

The application of virtual reality technology as an auxiliary tool in table tennis teaching is conducive to improving learners' interest in table tennis, allowing students to quickly enter their role in the process of participating in learning, to achieve the purpose of training and teaching, and to develop a sense of physical exercise and behavioral habits.

### 4.1. Consistency Analysis of Different Groups before the Experiment

#### 4.1.1. Consistency Analysis of Autonomous Learning Ability

Students' autonomous learning ability is based on the learners' acquisition of learning methods and skills in the learning process, determining learning goals, selecting learning content, monitoring the learning process, and evaluating the integrity of learning results. In order to explore whether there is a statistical difference between the control class and the experimental class in the autonomous learning ability of college students before the start of the table tennis course, a one-way analysis of variance was used to conduct a comparative analysis between different groups, as shown in Table 5.

The article "The Application of Virtual Reality Technology in Sports Psychology: Theory, Practice, and Prospect" was published in 2022. Journal: Comput Intell Neurosci.

According to the consistency analysis results of the autonomous learning ability of different groups, before the table tennis teaching experiment started, there was no significant difference between the control class and the experimental class in the autonomous learning ability (*F* = 0.368, *P* > 0.05). There is also no significant difference between the four dimensions of “learning motivation, learning process, learning result and learning environment” (*P* > 0.05). It shows that learners of different groups tend to be consistent in terms of self-learning ability, attitude, and cognition, which creates a prerequisite for the development of this research experiment.

#### 4.1.2. Consistency Analysis of Sports Situation Interests

In order to observe whether there is a statistical difference in the interest of college students in sports situations between the control class and the experimental class before the experiment, a one-way analysis of variance was used to compare and analyze the data of different groups, as shown in Table 6.

According to the consistency analysis results of different groups of sports situational interest, before the table tennis teaching experiment started, the sports situational interest of the students in the control class and the experimental class (*F* = 0.103, *P* > 0.05) and “novelty, challenge, attention.” There was no significant difference in the six dimensions of test content (*P* > 0.05). It shows that different groups of college students tend to have the same level of sports interest before participating in the table tennis course, which meets the requirements of teaching experiments.

### 4.2. Analysis of the Learning Effect of Virtual Reality Teaching

With the in-depth integration of virtual simulation technology and education, an immersive teaching scene is created for learners. Students use a variety of hardware devices to interact and feedback between humans and machines from a first-person perspective to enhance their learning experience. However, whether virtual reality teaching can promote the improvement of the table tennis teaching effect is still not an exact answer. In order to explore the potential value of VR in teaching, a paired sample *T*-test was used to make a longitudinal comparison of various test contents among 32 learners in the virtual reality teaching class, as shown in Table 7.

Through the analysis of the learning effect of virtual reality table tennis teaching, after the intervention of virtual reality sports games for a natural semester, the subjects in terms of autonomous learning ability, learning motivation (*T* = −4.158, *P* < 0.05), learning process (*T* = −2.502, *P* < 0.05), and learning results (*T* = −8.617, *P* < 0.05) were significantly different from those before the experiment. Description: based on the HTC Vive virtual reality device as an auxiliary teaching tool for table tennis elective courses in colleges and universities, it creates a highly immersive table tennis learning environment for participants with freedom of human-computer interaction, feedback in the practice process, and authenticity of virtual scenes. In the virtual situation of exploration, the intrinsic motivation of exercise is stimulated, and the space for students to think independently is given. However, there is no significant difference in the learning environment (*T* = 0.272, *P* = 0.787 > 0.05). According to the topic, the learning environment mainly revolves around giving students some free choice of activities in the classroom, while the learning environment is created by VR equipment. The virtual simulation teaching environment can fully guarantee the enthusiasm of students to explore, and the absence of differences in this indicator just reflects the superiority of VR teaching.

The article "The Application of Virtual Reality Technology in Sports Psychology: Theory, Practice, and Prospect" was published in 2022. Journal: Comput Intell Neurosci.

## 5. Conclusion

To sum up, the key of VR technology is to focus on the word “virtual.” Compared with reality, it is fictitious, but it is more real than pure imagination and traditional two-dimensional presentation. The development of science and technology has brought about an increase in the sense of immersion. It is believed that in the near future, people will experience sensory stimulation that is infinitely close to reality in the virtual environment. While psychology is a science that studies people, VR technology provides a new direction and method for us to understand, predict, and intervene in human behavior in real life, and get rid of the constraints of the real environment. This research applies virtual reality technology to the teaching of table tennis in colleges and universities. Through the analysis of the learning effect of virtual reality table tennis teaching, it is found that the learning environment created by VR equipment can fully guarantee the enthusiasm of students to explore, and the lack of difference in this indicator precisely reflects the superiority of VR teaching. Hence, the study presented in this article has good practical significance for the improvement of table tennis sports skills learning, autonomous learning ability, and learning interest of college students. Informatization transformation provides a practical basis.

## Figures and Tables

**Figure 1:** Human perception and generation of VR scenes.

The article "The Application of Virtual Reality Technology in Sports Psychology: Theory, Practice, and Prospect" was published in 2022. Journal: Comput Intell Neurosci.

**Figure 2:** Structure diagram of VR-based competitive sports simulation system.

**Figure 3:** VR perception interaction model.

**Figure 4:** Schematic diagram of forward kinetics.

**Figure 5:** Flowchart of motion capture technology implementation.

**Figure 6:** P3P iterative algorithm solution.

**Figure 7:** The specific implementation flow chart of the PNP algorithm.

**Table 1:** Distribution of countries that published relevant literature from 1995 to 2019 (top 10).

Rank	Number of documents (articles)	Nation
1	1041	USA
2	310	England
3	285	People's Republic of China
4	259	Germany
5	232	Spain
6	215	Canada
7	215	South Korea
8	206	Italy
9	156	Netherlands
10	150	France

**Table 2:** Basic information of research objects.

Basic situation	Traditional classes	Virtual reality class	Video teaching class
Grade	Class of 2018	Class of 2018	Class of 2018
Number of people	34	32	31
Profession	Social development and public administration	Art college	School of education

**Table 3:** Reliability test table.

Scale	Different dimension variables	Scale item	Cronbach's coefficient
College students' physical education self-learning scale	Motivation to learn	11	0.914
	Learning process	10	0.900
	Learning environment	6	0.707
	Learning outcomes	9	0.884

Sports situational interest scale	Novelty	4	0.715
	Challenge	4	0.748
	Attention	4	0.789
	Exploratory	4	0.753
	Pleasure	4	0.835
	General interest	4	0.848

**Table 4:** Validity test table.

Scale	Different dimension variables	Scale item	KMO	Bartlett approximate chi-square	Sphere test significance
College students' physical education self-learning scale	Motivation to learn	11	0.937	496.310	0.000
	Learning process	10	0.904	419.877	0.000
	Learning environment	6	0.758	89.661	0.000
	Learning outcomes	9	0.894	370.912	0.000

Sports situational interest scale	Novelty	4	0.705	109.114	0.000
	Challenge	4	0.723	111.509	0.000
	Attention	4	0.713	117.963	0.000
	Exploratory	4	0.750	94.062	0.000
	Pleasure	4	0.757	171.388	0.000
	General interest	4	0.779	181.377	0.000

**Table 5:** Consistency analysis of autonomous learning ability.

	Traditional classes		Virtual reality class		Video teaching class		*F*	*P*
	M	SD	M	SD	M	SD		
Motivation to learn	2.933	0.926	2.889	0.926	2.871	0.861	0.041	0.960
Learning process	2.827	0.853	2.781	0.924	3.026	0.857	0.691	0.504
Learning outcomes	3.154	0.877	2.826	1.149	2.760	0.634	1.759	0.178
Learning environment	3.177	0.712	3.135	0.624	3.011	0.676	0.526	0.592
Self-learning ability	2.999	0.576	2.885	0.606	2.910	0.531	0.368	0.693

Notes: ^*∗*^The significance level for the difference in means is 0.05. ^∗∗^The significance level for the difference in means is 0.01.

**Table 6:** Consistency analysis of sports situational interest.

	Traditional classes		Virtual reality class		Video teaching class		*F*	*P*
	M	SD	M	SD	M	SD		
Novelty	2.993	0.620	3.063	0.803	3.081	0.630	0.150	0.861
Challenge	2.882	0.613	2.883	0.765	2.758	0.572	0.381	0.684
Attention	2.463	0.600	2.570	0.554	2.500	0.555	0.297	0.744
Exploratory	2.559	0.511	2.617	0.568	2.565	0.536	0.115	0.891
Pleasure	2.963	0.677	2.836	0.834	3.024	0.634	0.563	0.571
General interest	2.868	0.497	2.734	0.770	2.621	0.686	1.147	0.300
Sports situational interest	2.788	0.222	2.784	0.374	2.758	0.235	0.103	0.902

Notes: ^*∗*^The significance level for the difference in means is 0.05. ^∗∗^The significance level for the difference in means is 0.01.

The article "The Application of Virtual Reality Technology in Sports Psychology: Theory, Practice, and Prospect" was published in 2022. Journal: Comput Intell Neurosci.

**Table 7:** Analysis of learning effect of virtual reality teaching class.

Test indicator	Pretest		Posttest		*T*	*P*
	M	SD	M	SD		
Motivation to learn	2.889	0.926	3.594	0.787	−4.158	0.000^∗∗∗^
Learning process	2.781	0.924	3.091	0.513	−2.502	0.018^*∗*^
Learning outcomes	2.826	1.149	3.938	0.502	−8.167	0.000^∗∗∗^
Learning environment	3.135	0.624	3.099	0.499	0.272	0.787
Self-learning ability	2.885	0.606	3.458	0.426	−7.990	0.000^∗∗∗^
Novelty	3.063	0.803	3.758	0.855	−2.94	0.000^∗∗∗^
Challenge	2.883	0.765	3.766	0.458	−5.632	0.000^∗∗∗^
Attention	2.57	0.554	3.102	0.605	−3.920	0.000^∗∗∗^
Exploratory	2.617	0.568	0.18	0.485	−3.552	0.000^∗∗∗^
Pleasure	2.836	0.834	0.547	0.455	−4.157	0.000^∗∗∗^
General interest	2.734	0.77	4.359	0.531	−9.966	0.000^∗∗∗^
Sports situational interest	2.784	0.374	3.619	0.281	−9.075	0.000^∗∗∗^
Forehand	7.281	2.303	12.625	2.624	−9.665	0.000^∗∗∗^
Two o'clock push a little	7.281	2.098	12.688	2.494	−14.616	0.000^∗∗∗^
Technical assessment score	3.156	1.139	6.469	1.135	−12.953	0.000^∗∗∗^
Skill assessment results	17.719	3.225	31.781	3.652	−19.314	0.000^∗∗∗^
50 m run	6.625	1.737	6.688	1.908	−0.203	0.840
Touch the ball table side by side	9.844	1.798	10.313	1.533	−1.305	0.201
Standing long jump	7.469	1.436	7.563	1.865	−0.237	0.814
Physical fitness	23.938	2.782	24.563	3.232	−1.232	0.227

Notes: ^*∗*^The significance level for the difference in means is 0.05. ^∗∗^The significance level for the difference in means is 0.01.

## Data Availability

The labeled data set used to support the findings of this study is available from the corresponding author upon request.
